The article "A Mathematical Model of COVID-19 with Vaccination and Treatment" was published in 2021. Journal: Comput Math Methods Med.

# A Mathematical Model of COVID-19 with Vaccination and Treatment

**DOI:** 10.1155/2021/1250129

**Published:** 2021-09-04

**Authors:** M. L. Diagne, H. Rwezaura, S. Y. Tchoumi, J. M. Tchuenche

**Affiliations:** ^1^Departement de Mathematiques, UFR des Sciences et Technologies, Universite de Thies, Thies, Senegal; ^2^Mathematics Department, University of Dar es Salaam, P.O. Box 35062, Dar es Salaam, Tanzania; ^3^Department of Mathematics and Computer Sciences ENSAI, University of Ngaoundere, P. O. Box 455 Ngaoundere, Cameroon; ^4^School of Computational and Communication Sciences and Engineering, Nelson Mandela African Institution of Science and Technology, P.O. Box 447, Arusha, Tanzania

## Abstract

We formulate and theoretically analyze a mathematical model of COVID-19 transmission mechanism incorporating vital dynamics of the disease and two key therapeutic measures—vaccination of susceptible individuals and recovery/treatment of infected individuals. Both the disease-free and endemic equilibrium are globally asymptotically stable when the effective reproduction number *R*_0_(*v*) is, respectively, less or greater than unity. The derived critical vaccination threshold is dependent on the vaccine efficacy for disease eradication whenever *R*_0_(*v*) > 1, even if vaccine coverage is high. Pontryagin's maximum principle is applied to establish the existence of the optimal control problem and to derive the necessary conditions to optimally mitigate the spread of the disease. The model is fitted with cumulative daily Senegal data, with a basic reproduction number *R*_0_ = 1.31 at the onset of the epidemic. Simulation results suggest that despite the effectiveness of COVID-19 vaccination and treatment to mitigate the spread of COVID-19, when *R*_0_(*v*) > 1, additional efforts such as nonpharmaceutical public health interventions should continue to be implemented. Using partial rank correlation coefficients and Latin hypercube sampling, sensitivity analysis is carried out to determine the relative importance of model parameters to disease transmission. Results shown graphically could help to inform the process of prioritizing public health intervention measures to be implemented and which model parameter to focus on in order to mitigate the spread of the disease. The effective contact rate *b*, the vaccine efficacy *ε*, the vaccination rate *v*, the fraction of exposed individuals who develop symptoms, and, respectively, the exit rates from the exposed and the asymptomatic classes *σ* and *ϕ* are the most impactful parameters.

## 1. Introduction

The December 2019 outbreak of the novel severe acute respiratory syndrome coronavirus 2 (SARS-CoV-2), causing COVID-19, was first reported in Wuhan, Hubei Province of China [1–4]. Coronaviruses can be extremely contagious and spread easily from person to person [5]. The disease, now a global pandemic, has spread rapidly worldwide, causing major public health concerns and economic crisis [3, 4, 6], having a massive impact on populations and economies and thereby placing an extra burden on health systems around the planet [7–9]. In fact, all social levels of the society have suffered major disruptions due to the COVID-19 pandemic [10].

The article "A Mathematical Model of COVID-19 with Vaccination and Treatment" was published in 2021. Journal: Comput Math Methods Med.

Starting with the work of Daniel Bernoulli in 1760 [11], the development of mathematical models has been critical in our understanding of the dynamics of infectious diseases [12]. With the work of Kermack and McKendrick [13], mathematical models have since been used to provide framework for understanding the dynamics of infectious diseases. COVID-19 transmission dynamics models are flourishing and abound in the literature [14–19], to cite a few and the references therein. With the availability of COVID-19 vaccine and its known high efficacy, there is an urgent need to assess the impact of such vaccines with imperfect transmission-blocking effects [6] and potentially refine previous mathematical models of COVID-19 that incorporated the potential impact of an imperfect vaccine [2, 8, 20]. A recent study by Pearson et al. [21] found that COVID-19 vaccination in low- and middle-income settings is highly cost-effective and even cost saving, when the vaccine is reasonably priced and efficacy is high. Prior to pharmaceutical measures such as treatment and vaccination being available, nonpharmaceutical intervention measures such as self-quarantine of confirmed cases, isolation, face masks, hand washing, social/physical distancing, and the most restrictive lockdowns, closure, or limited openings of shops and schools have been relied upon and continue to be widely implemented [22–24].

As COVID-19 vaccines are being deployed worldwide, we formulate and qualitatively analyze a COVID-19 mathematical model, taking into consideration available therapeutic measures, vaccination of susceptible and treatment of hospitalized/infected individuals. Our proposed model incorporates some key epidemiological and biological features of COVID-19, including demographic parameters (recruitment/birth and death). Optimal control is carried out using Pontryagin's maximum principle as described in [25] and applied in epidemiological models [26–35]. To identify the model parameters with greater influence on the initial disease transmission *R*_0_(*v*) when vaccination and treatment are implemented [36], a sensitivity analysis is carried out using partial rank correlation coefficients (PRCCs) and the results are shown graphically. This identification is crucial to inform policy decision on which parameters to focus either for data collection or to mitigate the spread of the disease. To the best of our knowledge, this study provides the first in-depth mathematical analysis of the qualitative dynamics of COVID-19 with an imperfect vaccine and treatment.

The article "A Mathematical Model of COVID-19 with Vaccination and Treatment" was published in 2021. Journal: Comput Math Methods Med.

The rest of the paper is organized as follows. The proposed COVID-19 model is formulated in Section 2 and theoretically analyzed in Section 3. By applying Pontryagin's maximum principle, optimal control of the model to mitigate the spread of COVID-19 is presented in Section 4. Numerical simulations performed to support theoretical results are presented in Section 5. The conclusion is provided in Section 6.

## 2. Model Formulation and Analysis

Consider a homogeneous mixing within the population, i.e., individuals in the population have equal probability of contact with each other. Using a deterministic compartmental modeling approach to describe the disease transmission dynamics, at any time *t*, the total population *N*(*t*) is subdivided into several epidemiological states depending on individuals' health status: susceptible *S*(*t*), vaccinated *V*(*t*), exposed *E*(*t*), symptomatic infected individuals *I*(*t*), infected asymptomatic *A*(*t*), hospitalized *H*(*t*), and recovered *R*(*t*). The total human population *N*(*t*) is given by

(1) $$\begin{array}{c} N\left(t\right)=S\left(t\right)+V\left(t\right)+E\left(t\right)+I\left(t\right)+A\left(t\right)+H\left(t\right)+R\left(t\right). \end{array}$$

Figure 1 depicts the schematic model flow. The description of the model variables and parameters is presented in Table 1.

Since COVID-19 vaccination is available, it is realistic to consider a specific vaccinated class *V*. The transition rates from susceptible and vaccinated to exposed is given by, respectively, by the following force of infection *β*_*S*_ = *b*((*ω*_*A*_*A* + *ω*_*I*_*I* + *ω*_*H*_*H*)/*N*) and *β*_*V*_ = (1 − *ε*)*β*_*S*_, where *b* is the effective contact rate, *ω*_*X*_ with *X* ∈ {*A*, *I*, *H*} represent the transmission probability after a contact with an individual in status *X*, and *ε* represents the infection reduction of vaccinated individuals. The nonlinearity of the force of infection is one of the key features of dynamic infectious disease models, because to model a population of individuals, the status of each individual is required [37]. Individuals are recruited into the population at a rate *Π*, with a fraction *p* vaccinated and the remaining (1 − *p*) susceptible. The latter are vaccinated at a rate *v*. Because vaccine could be imperfect, that is, vaccination providing only partial protection, we assume that vaccinated individuals can become exposed to the disease *b*(1 − *ε*). It has been shown that even a partially efficacious vaccine can offer a fundamental solution to the SARS-CoV-2 pandemic [20]. The parameter *ε* represents the vaccine efficacy (or infection reduction of vaccinated individuals).

The article "A Mathematical Model of COVID-19 with Vaccination and Treatment" was published in 2021. Journal: Comput Math Methods Med.

After close contacts with symptomatic, asymptomatic, and hospitalized individuals, susceptible become exposed with the disease. We assume that the rate of disease transmission from asymptomatic to susceptible individuals is less than that from symptomatic and hospitalized individuals. While outbreaks usually persist for a shorter period of time, the COVID-19 pandemic which started in December 2019 is still ongoing, and for this reason, we incorporate vital dynamics (recruitment and death). Let *σ* be the exit rate from exposed class where a fraction *ψ* develops infection while the remaining 1 − *ψ* becomes asymptomatic. The exit rate from the asymptomatic class is *λ*. Asymptomatic individuals *A* are diminished by natural death at a rate *μ* (it is assumed that death due to the disease in this group of individuals is negligible), by those developing symptoms and moving to the asymptomatic class at a rate (1 − *ϕ*), while a fraction *ϕ* may recover naturally from the asymptomatic infection and move to the recovered class *R*. Exit from the infected class is *γ*, where a fraction (1 − *κ*) are hospitalized, and a fraction *κ* recovers naturally. Finally, hospitalized individuals are treated and recovered at a rate *τ*. It is assumed that symptomatic and hospitalized individuals experience and additional disease-induced death rate *δ*, respectively. We also consider that the recovered individuals die at a rate *μ*, while a fraction *η* becomes susceptible again.

From the aforementioned and the model flow diagram of the disease transmission mechanisms Figure 1, we derive the following nonlinear system of ordinary differential equations that captures the transmission dynamics of COVID-19.

From the model flow diagram in Figure 1, we derive the following system of nonlinear ordinary differential equations:

(2) $$\begin{array}{c} \left\{\begin{array}{c} \dot{S}=\left(1-p\right)\Pi +\eta R-\left(\beta_{S}+\mu +v\right)S,\\ \dot{V}=p\Pi +vS-\left(\beta_{V}+\mu \right)V,\\ \dot{E}=\beta_{S}S+\beta_{V}V-\left(\sigma +\mu \right)E,\\ \dot{I}=\sigma \psi E+\lambda \left(1-\phi \right)A-\left(\gamma +\mu +\delta \right)I,\\ \dot{A}=\sigma \left(1-\psi \right)E-\left(\lambda +\mu \right)A,\\ \dot{H}=\gamma \left(1-\kappa \right)I-\left(\tau +\mu +\delta \right)H,\\ \dot{R}=\gamma \kappa I+\lambda \phi A+\tau H-\left(\eta +\mu \right)R, \end{array}\right. \end{array}$$

with initial conditions

(3) $$\begin{array}{c} S\left(0\right)\geq 0,\\ V\left(0\right)\geq 0,\\ \;E\left(0\right)\geq 0,\\ I\left(0\right)\geq 0,\\ \;A\left(0\right)\geq 0,\\ \;H\left(0\right)\geq 0,\\ \;R\left(0\right)\geq 0, \end{array}$$

where

(4) $$\begin{array}{c} \beta_{S}=b\frac{\omega_{A}A+\omega_{I}I+\omega_{H}H}{N},\\ \beta_{V}=b\left(1-\varepsilon \right)\frac{\omega_{A}A+\omega_{I}I+\omega_{H}H}{N}. \end{array}$$

For simplicity, let *g*_1_ = *μ* + *v*, *g*_2_ = *μ*, *g*_3_ = *σ* + *μ*, *g*_4_ = *γ* + *μ* + *δ*, *g*_5_ = *λ* + *μ*, *g*_6_ = *τ* + *μ* + *δ*, and *g*_7_ = (*η* + *μ*). Then, model system 1 now reads

(5) $$\begin{array}{c} \left\{\begin{array}{c} \dot{S}=\left(1-p\right)\Pi +\eta R-\left(\beta_{S}+g_{1}\right)S,\\ \dot{V}=p\Pi +vS-\left(\beta_{V}+g_{2}\right)V,\\ \dot{E}=\beta_{S}S+\beta_{V}V-g_{3}E,\\ \dot{I}=\sigma \psi E+\lambda \left(1-\phi \right)\text{A}-g_{4}I,\\ \dot{A}=\sigma \left(1-\psi \right)E-g_{5}A,\\ \dot{H}=\gamma \left(1-\kappa \right)I-g_{6}H,\\ \dot{R}=\gamma \kappa I+\lambda \phi A+\tau H-g_{7}R. \end{array}\right. \end{array}$$

All the model parameters and their description, values, and sources are presented in Table 1.

The article "A Mathematical Model of COVID-19 with Vaccination and Treatment" was published in 2021. Journal: Comput Math Methods Med.

## 3. Model Analysis

Well-posedness, nonnegativity, and boundedness of solutions of the proposed model can be shown using basic theory of dynamical systems as described in [43, 44]; also see [45, 46]. By adding all the equations of the system, we have $\dot{N}=\Pi -\mu N-\delta \left(I+H\right)\leq \Pi -\mu N$. Therefore, it follows that the biologically feasible region for model 1 is

(6) $$\begin{array}{c} D=\left\{\left(S,V,E,I,A,H,R\right)\in {\mathbb{R}}_{+}^{7}:N\leq \frac{\Pi }{\mu }\right\}. \end{array}$$

### 3.1. Disease-Free Equilibrium and Basic Reproduction Number

Model system 1 admits a disease-free equilibrium (DFE) given by *E*^0^ = (*S*^0^, *V*^0^, 0, 0, 0, 0, 0), where

(7) $$\begin{array}{c} S^{0}=\frac{\Pi \left(1-p\right)}{g_{1}},\\ V^{0}=\frac{\Pi \left[pg_{1}+v\left(1-p\right)\right]}{g_{1}g_{2}}. \end{array}$$

The linear stability of *E*^0^ is established using the next-generation method [47, 48]. The rate of appearance of new infections and the rate of transfer of individuals by all other means are given by the following at least twice continuously differentiable functions

(8) $$\begin{array}{c} F=\left[\begin{array}{c} b\frac{\omega_{A}A+\omega_{I}I+\omega_{H}H}{N}S+b\left(1-\varepsilon \right)\frac{\omega_{A}A+\omega_{I}I+\omega_{H}H}{N}V\\ 0\\ 0\\ 0 \end{array}\right],\\ V=\left[\begin{array}{c} -g_{3}E\\ \sigma \psi E+\lambda \left(1-\phi \right)A-g_{4}I\\ \sigma \left(1-\psi \right)E-g_{5}A\\ \gamma \left(1-\kappa \right)I-g_{6}H \end{array}\right]. \end{array}$$

From [48], the nonnegative matrix *F* and the nonsingular *M*-matrix *V* for the new infection terms and the remaining transfer terms are given by

(9) $$\begin{array}{c} F=\left[\begin{array}{cccc} 0 & \frac{b\omega_{I}\left(S^{0}+\left(1-\varepsilon \right)V^{0}\right)}{N^{0}} & \frac{b\omega_{A}\left(S^{0}+\left(1-\varepsilon \right)V^{0}\right)}{N^{0}} & \frac{b\omega_{H}\left(S^{0}+\left(1-\varepsilon \right)V^{0}\right)}{N^{0}}\\ 0 & 0 & 0 & 0\\ 0 & 0 & 0 & 0\\ 0 & 0 & 0 & 0 \end{array}\right],\\ V=\left[\begin{array}{cccc} -g_{3} & 0 & 0 & 0\\ \sigma \psi & -g_{4} & \lambda \left(1-\phi \right) & 0\\ \sigma \left(1-\psi \right) & 0 & -g_{5} & 0\\ 0 & \gamma \left(1-\kappa \right) & 0 & -g_{6} \end{array}\right]. \end{array}$$

Thus, the effective reproduction number is given by

(10) $$\begin{array}{c} R_{0}\left(v\right)=\frac{\left[\left(\lambda \left(1-\phi \right)\left(1-\psi \right)+g_{5}\psi \right)\left(g_{6}\omega_{I}+\gamma \left(1-\kappa \right)\omega_{H}\right)+g_{4}g_{6}\left(1-\psi \right)\omega_{A}\right]\left[g_{2}\left(1-p\right)+\left(1-\varepsilon \right)\left(pg_{1}+\left(1-p\right)v\right)\right]b\mu \sigma }{g_{1}g_{2}g_{3}g_{4}g_{5}g_{6}}=\frac{b\mu \sigma \left[G_{1}G_{2}+G_{3}\right]\left[G_{4}+\left(1-\varepsilon \right)\left(p\left(\mu +v\right)+\left(1-p\right)v\right)\right]}{\left(\mu +v\right)g_{2}g_{3}g_{4}g_{5}g_{6}}, \end{array}$$

where *G*_1_ = ((*λ*(1 − *ϕ*)(1 − *ψ*) + *g*_5_*ψ*), *G*_2_ = (*g*_6_*ω*_*I*_ + *γ*(1 − *κ*)*ω*_*H*_), *G*_3_ = *g*_4_*g*_6_(1 − *ψ*)*ω*_*A*_, and *G*_4_ = *g*_2_(1 − *p*).

The article "A Mathematical Model of COVID-19 with Vaccination and Treatment" was published in 2021. Journal: Comput Math Methods Med.

The effective reproduction number *R*_0_(*v*) is defined as the average number of secondary infections generated by a single infectious individual during his entire duration infectiousness in a totally susceptible population when vaccination is implemented.

### 3.2. Stability of the Disease-Free Equilibrium

We now study the global stability of the DFE using the approach described in [49]. Consider a system of ordinary differential equations of the form

(11) $$\begin{array}{c} \left\{\begin{array}{c} \frac{dx}{dt}=F\left(x,I\right),\\ \frac{dI}{dt}=G\left(x,I\right),G\left(x,0\right)=0, \end{array}\right. \end{array}$$

where *x* ∈ ℝ^*m*^ denotes (its components) the number of uninfected individuals and *I* ∈ ℝ^*n*^ denotes (its components) the number of infected individuals including latent and infectious. Let *U*_0_ = (*x*^∗^, 0) be the disease-free equilibrium of this system, where 0 is a zero vector. Global stability of the DFE is guaranteed when the following conditions (H1) and (H2) are satisfied.

The article "A Mathematical Model of COVID-19 with Vaccination and Treatment" was published in 2021. Journal: Comput Math Methods Med.

(H1) For *dx*/*dt* = *F*(*x*, 0), 0 is globally asymptotically stable (g.a.s.).

(H2) $G\left(x,I\right)=AI-\hat{G}\left(x,I\right),\;\hat{G}\left(x,I\right)⩾0$ for (*x*, *I*) ∈ *Ω*, where *A* = *D*_*I*_*G*(*x*^∗^, 0) is an *M*-matrix (the off diagonal elements of *A* are nonnegative) and *Ω* is the region where the model makes biological sense.

**Corollary 1 (see [49]).**

The fixed point *U*_0_ = (*x*^∗^, 0) is a globally asymptotic stable (g.a.s.) equilibrium of (11) provided that *R*_0_(*v*) < 1 (l.a.s.) and that assumptions (H1) and (H2) are satisfied.

**Theorem 1 (global asymptotic stability of the DFE).**

The DFE *E*_0_ of model 1 is globally asymptotically stable if *R*_0_(*v*) < 1.

**Proof**

First, we rewrite model 1 in the form 6 by setting *x* = (*S*, *V*) and *I* = (*E*, *I*, *A*, *H*, *R*).

Then, the DFE is given by *U*_0_ = (*x*^∗^, 0) = (*Π*(1 − *p*)/*g*_1_, (*Π*[*pg*_1_ + *v*(1 − *p*)])/*g*_1_*g*_2_, 0) and the system *dx*/*dt* = *F*(*x*, 0) becomes

(12) $$\begin{array}{c} \left\{\begin{array}{c} \dot{S}=\left(1-p\right)\Pi -g_{1}S,\\ \dot{V}=p\Pi +vS-g_{2}V. \end{array}\right. \end{array}$$

This equation has a unique equilibrium point

(13) $$\begin{array}{c} x^{*}=\left(\frac{\Pi \left(1-p\right)}{g_{1}},\;\frac{\Pi \left[pg_{1}+v\left(1-p\right)\right]}{g_{1}g_{2}}\right), \end{array}$$

which is globally asymptotically stable. Therefore, the condition (H1) is satisfied.

We now verify the second condition (H2). For model 1, we have

(14) $$\begin{array}{c} G\left(x,I\right)=\left(\begin{array}{c} \beta_{S}S+\beta_{V}V-g_{3}E\\ \sigma \psi E+\lambda \left(1-\phi \right)A-g_{4}I\\ \sigma \left(1-\psi \right)E-g_{5}A\\ \gamma \left(1-\kappa \right)I-g_{6}H\\ \gamma \kappa I+\lambda \phi A+\tau H-g_{7}R \end{array}\right), \end{array}$$

(15) $$\begin{array}{c} D_{I}G\left(x^{*},0\right)=\left(\begin{array}{ccccc} -g_{3} & \frac{b\omega_{I}}{N^{0}}\left(S^{0}+V^{0}\left(1-\varepsilon \right)\right) & \frac{b\omega_{A}}{N^{0}}\left(S^{0}+V^{0}\left(1-\varepsilon \right)\right) & \frac{b\omega_{H}}{N^{0}}\left(S^{0}+V^{0}\left(1-\varepsilon \right)\right) & 0\\ \sigma \psi & -g_{4} & \lambda \left(1-\Phi \right) & 0 & 0\\ \sigma \left(1-\psi \right) & 0 & -g_{5} & 0 & 0\\ 0 & \gamma \left(1-\kappa \right) & 0 & -g_{6} & 0\\ 0 & \gamma \kappa & \lambda \Phi & 0 & -g_{7} \end{array}\right). \end{array}$$

Clearly, *A* is an *M*-matrix. On the other hand,

(16) $$\begin{array}{c} \hat{G}\left(x,I\right)=AI-G\left(x,I\right)=\left(\begin{array}{c} \beta_{S}\left(\frac{S^{0}}{N^{0}}-S\right)+\beta_{v}\left(\frac{V^{0}}{N^{0}}-V\right)\\ 0\\ 0\\ 0\\ 0 \end{array}\right), \end{array}$$

which implies that $\hat{G}\left(x,I\right)⩾0$ for all (*x*, *I*) ∈ *Ω*. Therefore, the conditions (H1) and (H2) are satisfied. By Corollary 1, the global stability of the DFE is obtained. This completes the proof.☐☐

Global stability of the DFE precludes the model to exhibit bistability also known as backward bifurcation [50, 51], a situation where both the disease-free and endemic equilibria coexist when *R*_0_(*v*) < 1.

The article "A Mathematical Model of COVID-19 with Vaccination and Treatment" was published in 2021. Journal: Comput Math Methods Med.

### 3.3. The Critical Vaccination Coverage

We investigate the critical vaccination coverage rate that could help eradicate the disease. *R*_0_(*v*)≔*ℛ*_*E*_. When there is no vaccination in the community, that is, *v* = 0, then the effective reproduction number reduces to

(17) $$\begin{array}{c} R_{0}=R_{0}\left(0\right)=\frac{b\sigma \left[G_{1}G_{2}+G_{3}\right]\left[G_{4}+\left(1-\varepsilon \right)p\mu \right]}{g_{2}g_{3}g_{4}g_{5}g_{6}}. \end{array}$$

In fact, *ℛ*_0_ is the so-called basic reproduction number which is the average number of secondary cases arising from one infectious individual in a totally susceptible population [47, 52]. After some rearrangement, *R*_0_(*v*) can be written as

(18) $$\begin{array}{c} R_{0}\left(v\right)=\frac{\mu }{\mu +v}\frac{G_{4}+\left(1-\varepsilon \right)\left(p\mu +v\right)}{G_{4}+\left(1-\varepsilon \right)p\mu }R_{0}=\frac{\mu }{\mu +v}\frac{\mu \left(1-p\right)+\left(1-\varepsilon \right)\left(p\mu +v\right)}{\mu \left(1-p\right)+\left(1-\varepsilon \right)p\mu }R_{0}=\frac{1}{\mu +v}\frac{\mu \left(1-\varepsilon p\right)+\left(1-\varepsilon \right)v}{\left(1-\varepsilon p\right)}R_{0}=\frac{R_{0}}{\mu +v}\left[\mu +\frac{\left(1-\varepsilon \right)v}{\left(1-\varepsilon p\right)}\right]=R_{0}\left[\frac{\mu }{\left(\mu +v\right)}+\frac{\left(1-\varepsilon \right)}{\left(1-\varepsilon p\right)}\frac{v}{\left(\mu +v\right)}\right]. \end{array}$$

Thus,

(19) $$\begin{array}{c} R_{0}\left(\infty \right)≔\underset{v⟶+\infty }{\lim}R_{0}\left(v\right)=\frac{\left(1-\varepsilon \right)}{\left(1-\varepsilon p\right)}R_{0}. \end{array}$$

Taking the partial derivative of *R*_0_(*v*) with respect to *v* yields

(20) $$\begin{array}{c} \begin{array}{c} \frac{\partial R_{0}\left(v\right)}{\partial v}=\frac{\mu }{{\left(\mu +v\right)}^{2}}\left[\frac{\varepsilon \left(p-1\right)}{\left(1-\varepsilon p\right)}\right]R_{0} \end{array}=-\frac{\varepsilon \left(1-p\right)}{\left(1-\varepsilon p\right)}\frac{\mu R_{0}}{{\left(\mu +v\right)}^{2}}<0. \end{array}$$

Therefore, ((1 − *ε*)/(1 − *εp*))*ℛ*_0_ ⩽ *R*_0_(*v*) ⩽ *ℛ*_0_, and hence, *ℛ*_0_ < 1 implies *R*_0_(*v*) < 1, but the reverse is not true. For *ℛ*_0_ > 1, it is important to note that

(21) $$\begin{array}{c} R_{0}\left(\infty \right)<1\Leftrightarrow \frac{\left(1-\varepsilon \right)}{\left(1-\varepsilon p\right)}R_{0}<1\Leftrightarrow \varepsilon >\varepsilon^{*}≔\frac{R_{0}-1}{R_{0}-p}. \end{array}$$

This can be interpreted to mean that when the vaccine efficacy *ε* is low and *ℛ*_0_ is far greater than unity, the disease may not be eradicated even if the vaccine coverage is high.  Figure 2 can be interpreted as additional efforts will be needed to reduce *R*_0_(*v*) below unity even when there is a high vaccine coverage *v*. In fact, the role of human/social behavior among those vaccinated (behavior compensation) such as careless increase in social/physical contacts can undermine vaccine impact [18, 20]. Thus, cautious phased relaxation of nonpharmaceutical interventions could substantially reduce population-level morbidity and mortality [23].

The article "A Mathematical Model of COVID-19 with Vaccination and Treatment" was published in 2021. Journal: Comput Math Methods Med.

The next result provides the critical vaccination threshold *v*^∗^ for disease eradication.

**Lemma 1 .**

Assume that the basic reproduction number *ℛ*_0_ > 1. Then, there exists

(22) $$\begin{array}{c} v^{*}=\frac{\mu \left(1-\varepsilon p\right)\left(R_{0}-1\right)}{\left(\varepsilon -\varepsilon^{*}\right)\left(R_{0}-p\right)}>0, \end{array}$$

such that *R*_0_(*v*^∗^) = 1. Furthermore, *R*_0_(*v*) > (<)1 when *v* < (>)*v*^∗^.

Figure 3 depicts the vaccine coverage *v* as a function of *ℛ*_0_, with a 91% vaccine efficacy (*ε* > *ε*^∗^). The green surface represents the case when the vaccine coverage *v* exceeds the critical vaccination threshold *v*^∗^.

### 3.4. Stability of the Endemic Equilibrium

After some algebraic manipulations, the endemic equilibrium of model system 1 is obtained as

(23) $$\begin{array}{c} S^{*}=\frac{\left(1-p\right)\Pi +\eta R^{*}}{\beta_{S}^{*}+g_{1}},\\ V^{*}=\frac{p\Pi +vS^{*}}{\left(1-\varepsilon \right)\beta_{S}^{*}+g_{2}},\\ E^{*}=\frac{\beta_{S}^{*}\left[S^{*}+\left(1-\varepsilon \right)V^{*}\right]}{g_{3}},\\ A^{*}=\frac{\sigma \left(1-\psi \right)E^{*}}{g_{5}},\\ I^{*}=\frac{\sigma \psi E^{*}+\lambda \left(1-\phi \right)A^{*}}{g_{4}},\\ H^{*}=\frac{\gamma \left(1-\kappa \right)I^{*}}{g_{6}}. \end{array}$$

From the last equation of model system 1 and using the definition of *β*_*S*_^∗^, we obtain the following quadratic equation

(24) $$\begin{array}{c} \beta_{S}^{*}\left[P_{2}\beta_{S}^{*2}+P_{1}\beta_{S}^{*}+P_{0}\right]=0, \end{array}$$

where *P*_1_ and *P*_2_ are positive constants given in the appendix and

(25) $$\begin{array}{c} P_{0}=g_{1}g_{2}g_{3}g_{4}g_{5}g_{6}\left(R_{0}\left(v\right)-1\right). \end{array}$$

Thus, *β*_*S*_^∗^ = 0 implies *I* = 0, which represents the disease-free equilibrium, and hence, because *P*_1_ and *P*_2_ are positive, equation (24) has a unique positive solution if and only if *P*_0_ > 0, which is fulfilled when *R*_0_(*v*) > 1. Therefore, we have the following result.

The article "A Mathematical Model of COVID-19 with Vaccination and Treatment" was published in 2021. Journal: Comput Math Methods Med.

**Lemma 2 .**

If *R*_0_(*v*) > 1, model system 1 has a unique endemic equilibrium *E*^∗^.

It can also be shown using the theory or permanence as described in [53] that when *R*_0_(*v*) > 1, the disease class *I*(*t*) is uniformly persistent, that is, there exists a positive constant *k*, such that

(26) $$\begin{array}{c} \lim\underset{t⟶\infty }{\inf}I\left(t\right)\geq k. \end{array}$$

Consequently, the model system is uniformly persistent when *R*_0_(*v*) > 1.

Figure 4 depicts the impact of the reduction in transmission from asymptomatic *ω*_*A*_, and the increase in transmission from symptomatic *ω*_*I*_ on the effective reproduction number *R*_0_(*v*) > 1 is shown in Figure 4. Similar graphical representation for different model parameters space can be found in [54]. The white panel in Figure 4 shows the endemic equilibrium regions in the (*ω*_*I*_, *ω*_*A*_) space when *R*_0_(*v*) > 1. The solid line corresponds to *R*_0_(*v*) = 1. To mitigate the spread of the disease, it is important that the reduction in the transmission from asymptomatic *ω*_*A*_ < 0.36 and the increase in transmission from symptomatic *ω*_*I*_ < 1.16.

## 4. Optimal Control Problem

We investigate the impact of implementing pharmaceutical interventions to mitigate the spread of COVID-19. To accomplish this, we introduce a set of time-dependent control variables (*u*_1_(*t*), *u*_2_(*t*) where

- *u*_1_(*t*) represents the implementation of continuous vaccination
- *u*_2_(*t*) represents treatment of infected (often hospitalized) individuals

The proposed COVID-19 model with optimal control (*u*_1_(*t*), *u*_2_(*t*)) consists of the following nonautonomous system of nonlinear ordinary differential equations.

(27) $$\begin{array}{c} \left\{\begin{array}{c} \dot{S}=\left(1-p\right)\Pi +\eta R-\left(\beta_{S}+\mu +u_{1}\right)S,\\ \dot{V}=p\Pi +u_{1}S-\left(\beta_{V}+\mu +u\right)V,\\ \dot{E}=\beta_{S}S+\beta_{V}V-\left(\sigma +\mu \right)E,\\ \dot{I}=\sigma \psi E+\lambda \left(1-\phi \right)A-\left(\gamma +\mu +\delta \right)I,\\ \dot{A}=\sigma \left(1-\psi \right)E-\left(\lambda +\mu \right)A,\\ \dot{H}=\gamma \left(1-\kappa \right)I-\left(u_{2}+\mu +\delta \right)H,\\ \dot{R}=\gamma \kappa I+\lambda \phi A+u_{2}H-\left(\eta +\mu \right)R. \end{array}\right. \end{array}$$

We wish to find the controls that minimize the total infected individuals, that is, to find an optimal control for the two control strategies while reducing their relative costs. In other words, we want to find the optimal values of (*u*_1_(*t*), *u*_2_(*t*)) that minimize the objective functional *J*(*u*_1_, *u*_2_) where

(28) $$\begin{array}{c} J\left(u_{1},u_{2}\right)=\int_{0}^{T}\left(A_{1}E+A_{2}I+A_{3}A+A_{4}H+B_{1}u_{1}^{2}\left(t\right)+B_{2}u_{2}^{2}\left(t\right)\right)dt, \end{array}$$

subject to the differential equation (27), where *T* is the final time. This objective functional involves the total exposed, asymptomatic, infected, and hospitalized individuals, along with the cost of applying the controls *u*_1_(*t*) and *u*_2_(*t*). We consider a quadratic objective functional for measuring the control cost as frequently used in the literature [29–32, 55]. The positive coefficients *A*_1_, *A*_2_, *A*_3_, *A*_4_, *B*_1_ and *B*_2_ are balancing weight parameters, while the controls (*u*_1_(*t*) and *u*_2_(*t*)) are bounded, Lebesgue integrable functions [31, 32]. We then seek to find optimal controls *u*_1_^∗^ and *u*_2_^∗^, such that

(29) $$\begin{array}{c} J\left(u_{1}^{*},u_{2}^{*}\right)=\underset{\Omega }{\min}J\left(u_{1},u_{2}\right). \end{array}$$

To derive the necessary conditions that the two optimal controls and corresponding states must satisfy, we apply Theorem 5.1 (Pontryagin's maximum principle [25]) in Fleming and Rishel [56] to develop the optimal system for which the necessary conditions that must be satisfied by an optimal control and its corresponding states are derived. In fact, Theorem 1 in Agusto [26] which is based on the boundedness of solution of model system 1 without control variables ensures the existence of the optimal control while the existence of an optimal control with a given control pair follows from Fleming and Rishel [56] and Caratheodory's existence theorem [57]. For discussions on various forms of the objective functional (linear, quadratic), see [30, 58].

(30) $$\begin{array}{c} ℍ=A_{1}E+A_{2}I+A_{3}A+A_{4}H+B_{1}u_{1}^{2}+B_{2}u_{2}^{2}+\xi_{1}\left[\left(1-p\right)\Pi +\eta R-\left(\beta_{S}+\mu +u_{1}\right)S\right]+\xi_{2}\left[p\Pi +u_{1}S-\left(\beta_{V}+\mu +u\right)V\right]+\xi_{3}\left[\beta_{S}S+\beta_{V}V-\left(\sigma +\mu \right)E\right]+\xi_{4}\left[\sigma \psi E+\lambda \left(1-\phi \right)A-\left(\gamma +\mu +\delta \right)I\right]+\xi_{5}\left[\sigma \left(1-\psi \right)E-\left(\lambda +\mu \right)A\right]+\xi_{6}\left[\gamma \left(1-\kappa \right)I-\left(u_{2}+\mu +\delta \right)H\right]+\xi_{7}\left[\gamma \kappa I+\lambda \phi A+u_{2}H-\left(\eta +\mu \right)R\right], \end{array}$$

where *ξ*_*i*_, *i* = 1, ⋯, 7 are the adjoint variables or costate variables. The following result presents the adjoint system and control characterization.

The article "A Mathematical Model of COVID-19 with Vaccination and Treatment" was published in 2021. Journal: Comput Math Methods Med.

**Theorem 2 .**

Given an optimal control (*u*_1_^∗^, *u*_2_^∗^) and corresponding state solutions (*S*, *V*, *E*, *I*, *A*, *H*, *R*) of the corresponding state system 1, there exists adjoint variables, *ξ*_*i*_, *i* = 1, ⋯, 7, satisfying

(31) $$\begin{array}{c} \left\{\begin{array}{c} \xi \prime_{1}=\left(1-\frac{S}{N}\right)\beta_{s}\left(\xi_{1}-\xi_{3}\right)+\frac{V}{N}\beta_{v}\left(\xi_{3}-\xi_{2}\right)+u_{1}\left(\xi_{1}-\xi_{2}\right)+\mu \xi_{1},\\ \xi \prime_{2}=\frac{\beta_{s}}{N}S\left(\xi_{3}-\xi_{1}\right)+\left(1-\frac{V}{N}\right)\beta_{v}\left(\xi_{3}-\xi_{2}\right)+u\left(\xi_{2}-\xi_{1}\right)+\mu \xi_{2},\\ \xi \prime_{3}=\frac{\beta_{s}}{N}S\left(\xi_{3}-\xi_{1}\right)+\frac{\beta_{v}}{N}V\left(\xi_{3}-\xi_{2}\right)+\sigma \phi \left(\xi_{5}-\xi_{4}\right)+\sigma \left(\xi_{3}-\xi_{5}\right)+\mu \xi_{3}-A_{1},\\ \xi \prime_{4}=\frac{S}{N}\left(\beta_{s}-b\omega_{I}\right)\left(\xi_{3}-\xi_{1}\right)+\frac{V}{N}\left(\beta_{v}-b\left(1-\varepsilon \right)\omega_{I}\right)\left(\xi_{3}-\xi_{2}\right)+\gamma \kappa \left(\xi_{6}-\xi_{7}\right)+\gamma \left(\xi_{4}-\xi_{6}\right)+\left(\mu +\delta \right)\xi_{4}-A_{2},\\ \xi \prime_{5}=\frac{S}{N}\left(\beta_{s}-b\omega_{A}\right)\left(\xi_{3}-\xi_{1}\right)\frac{V}{N}\left(\beta_{v}-b\left(1-\varepsilon \right)\omega_{A}\right)\left(\xi_{3}-\xi_{2}\right)+\Phi \lambda \left(\xi_{4}-\xi_{7}\right)+\lambda \left(\xi_{5}-\xi_{4}\right)+\mu \xi_{5}-A_{3},\\ \xi \prime_{6}=\frac{S}{N}\left(b\omega_{H}-\beta_{s}\right)\left(\xi_{1}-\xi_{3}\right)+\frac{V}{N}\left(b\left(1-\varepsilon \right)-\beta_{v}\right)\left(\xi_{2}-\xi_{3}\right)+u_{2}\left(\xi_{6}-\xi_{7}\right)+\left(\mu +\delta \right)\xi_{6}-A_{4},\\ \xi \prime_{7}=\frac{S}{N}\left(\xi_{3}-\xi_{1}\right)+\frac{V}{N}\beta_{v}\left(\xi_{3}-\xi_{2}\right)+\eta \left(\xi_{7}-\xi_{1}\right)+\mu \xi_{7},\\ \xi \prime_{i}\left(T\right)=0\;\text{for}\;i=1,\cdots 7. \end{array}\right. \end{array}$$

The controls *u*_1_^∗^ and *u*_2_^∗^ satisfy the following optimality condition:

(32) $$\begin{array}{c} \left\{\begin{array}{c} u_{1}^{*}=\max\left\{0,\min\left(1,\frac{\left(\xi_{2}-\xi_{1}\right)S}{2B_{1}}\right)\right\},\\ u_{2}^{*}=\max\left\{0,\min\left(1,\frac{\left(\xi_{7}-\xi_{6}\right)H}{2B_{2}}\right)\right\}, \end{array}\right. \end{array}$$

**Proof**

The differential equations governing the adjoint variables are obtained by differentiation of the Hamiltonian function, evaluated at the optimal control. Then, the adjoint system can be written as

(33) $$\begin{array}{c} \begin{array}{c} \xi \prime_{1}=-\frac{\partial ℍ}{\partial S}, \end{array}\\ \xi \prime_{2}=-\frac{\partial ℍ}{\partial V},\\ \xi \prime_{3}=-\frac{\partial ℍ}{\partial E},\\ \xi \prime_{4}=-\frac{\partial ℍ}{\partial I},\\ \xi_{5}^{\prime }=-\frac{\partial ℍ}{\partial A},\\ \xi \prime_{6}=-\frac{\partial ℍ}{\partial H},\\ \xi \prime_{7}=-\frac{\partial ℍ}{\partial R}, \end{array}$$

with zero final time conditions (transversality) *ξ*_*i*_(*T*) = 0. Replacing the derivatives of *ℍ* with respect to *S*, *V*, *E*, *I*, *A*, *H*, *R* in the above equations, we obtain the optimality condition (32). The optimal conditions for the Hamiltonian are given by *∂ℍ*/*∂u*_1_^∗^ = *∂ℍ*/*∂u*_2_^∗^ = 0 or equivalently *∂ℍ*/*∂u*_1_^∗^ = 2*B*_1_*u*_1_^∗^ + (*ξ*_2_ − *ξ*_1_)*S* = 0, *∂ℍ*/*∂u*_2_^∗^ = 2*B*_2_*u*_2_^∗^ + (*ξ*_7_ − *ξ*_6_)*H* = 0.From the above equations, we obtain

(34) $$\begin{array}{c} u_{1}^{*}=\frac{\left(\xi_{1}-\xi_{2}\right)S}{2B_{1}},\\ u_{2}^{*}=\frac{\left(\xi_{6}-\xi_{7}\right)H}{2B_{2}}. \end{array}$$

Thus, *u*_1_^∗^ and *u*_2_^∗^ satisfy (32).☐☐

The article "A Mathematical Model of COVID-19 with Vaccination and Treatment" was published in 2021. Journal: Comput Math Methods Med.

## 5. Numerical Simulations

To illustrate the theoretical results, numerical simulations are carried out. Model parameter values for the numerical simulations with their description and source are listed in Table 1. Whenever parameter values were not available in the literature, we assumed realistic values for the purpose of illustration.

### 5.1. Model Fitting

Following the approach described in [14], model system 1 is fitted with daily new COVID-19 cases in Senegal from 29 March to 29 April 2020, which correspond to the first wave of infections in the country. It is important to note that while starting with an expanded model helps to account for the various disease classes explicitly, for the model fitting, model system 1 is reduced to a simpler version which retains the key compartments and characteristics of the complex one by eliminating similar classes [28]. This reduction involves removing the asymptomatic and hospitalized classes, which implies that the reduction in the transmission from hospitalized individuals is equated to zero, that is, *ω*_*H*_ = 0. The main key requirement for the simple model to approximate the complex one is that the susceptible class *S* should contain the same number of individuals in both models (when one compares both models compartment wise). The observed data were fitted in MatLab using the optimization function *createOptimProblem*. The estimated value of the basic reproduction number of the disease in Senegal during the period under consideration is *R*_0_ = 1.31, a value close to unity, which might explain why the first wave of COVID-19 infections did not pick up in Senegal.  Figure 5 depicts the daily cumulative number of COVID-19 cases in Senegal. Red dots represent actual confirmed cases while the blue curve is the best fitting curve of the model.

### 5.2. Long-Term Dynamics of the Disease

We investigated the impact of vaccination and treatment on mitigating the spread of COVID-19. An iterative fourth-order Runge-Kutta method (both forward and backward algorithms) is employed to compute the optimal controls and state values used. For more details on this approach, see [29, 32].

The article "A Mathematical Model of COVID-19 with Vaccination and Treatment" was published in 2021. Journal: Comput Math Methods Med.

The baseline weight parameters *A*_1_ = *A*_2_ = *A*_3_ = *A*_4_ = 1, *B*_1_ = 12, *B*_2_ = 19 are chosen to illustrate the optimal control strategies, as well as the following nonnegative initial conditions *S* = 2500, *V* = 10, *E* = 20, *I* = 70, *A* = 3, *H* = 3, *R* = 1. These weights do not necessarily have a significant meaning attached, but are only of theoretical sense to illustrate our proposed control strategies [31–33, 59]. Using parameter values in Table 1, the reproduction number *R*_0_(*v*) > 1, indicating that the disease is endemic in the population. The positive constants *A*_1_, *A*_2_, *A*_3_, and *A*_4_ represent, respectively, the weight that balance off the COVID-19 exposed, infected, asymptomatic, and hospitalized individuals; *B*_1_ and *B*_2_ are, respectively, the weight constant for vaccination and treatment. Because low cost could potentially be associated with COVID-19 vaccination compared to its treatment (as the cost associated to *u*_2_(*t*) includes the cost of medical examination, hospitalization, and medicines), the weight factor *B*_1_ has been made lower than *B*_2_, while the two control strategies *u*_1_, *u*_2_ are all constrained between zero and one, that is, 0 ≤ *u*_*i*_(*t*) ≤ 1, *i* = 1, 2. For instance, if *u*_1_ = 0, it implies no COVID-19 vaccination, and *u*_1_ ≠ 0 implies vaccination campaign measures are being implemented in the community. Table 1 provides all the model parameter values used for the simulations.

Figure 6 depicts the time series of model system 1 for the susceptible, vaccinated, exposed, and infected classes. Because of the potential limitations of vaccines in some settings, we consider in Figure 7 a saturated Holling type II vaccination rate

(35) $$\begin{array}{c} v≔\frac{v}{1+\xi S}, \end{array}$$

where *ξ* represents the limitation of the availability of vaccine [60]. We observe that when vaccines are widely available, the number of susceptible individuals decreases pretty fast as more and more people are getting the vaccine (the vaccinated class *V* increases at the onset of implementation (Figure 7)).

### 5.3. Impact of Control Interventions: Vaccination and Treatment

In the next set of figures generated from model system 14, optimal control strategies are implemented. Using the model parameter values in Table 1, the basic reproduction number *ℛ*_0_ = 2.21 > 1. For community with no vaccination program (*v* = 0), the basic reproduction number *ℛ*_0_ = 4.67 is almost double compared to the case when vaccination program is introduced. These values are in agreement with those estimated in recent COVID-19 modeling studies [61–63]. Figures 8–12 depict the graphical representations of the simulations of the COVID-19 model as a function of time without control and with optimal control. As can be observed on Figures 8–12, implementing control measures at the optimum level could help to mitigate the spread of the disease as shown by the significant decrease in the total number of individuals in the diseased classes and an increased in the vaccinated class.  Figure 13 depicts the profile for the effect of the control functions *u*_1_(*t*) and *u*_2_(*t*) on the dynamics of the model system. The two control measures need to be optimally implemented for the first 75 days and maintained for at least 3 months (close to 100 days). It is important however to note that while therapeutic measures, vaccination, and treatment are very effective in curtailing the spread of the epidemic, more control efforts are required to eradicate the disease when *R*_0_(*v*) > 1. Thus, continuously and concurrently applying both pharmaceutical and nonpharmaceutical public health interventions such as face mask, hand washing, and social distancing should be encouraged [64].

The article "A Mathematical Model of COVID-19 with Vaccination and Treatment" was published in 2021. Journal: Comput Math Methods Med.

### 5.4. Sensitivity of the Reproduction Number *R*_0_(*v*)

Because mathematical models are symbolic/mechanistic representations of complex biological systems, some model parameter values are not often known with certainty due to natural and seasonal variations, potential measurement errors [18]. To show how changes in model parameters values affect *R*_0_(*v*), we determine the relative importance of model parameters to disease transmission and graphically depict how sensitive the effective reproduction number is to the model parameters. Early ranking the intervention measures and other model parameters based on their impact could ideally partially inform the process of prioritizing public health intervention measures to be implemented, thereby helping policy and decision-makers to focus on those key impactful interventions.  Figure 14 indicates that when the vaccine efficacy *ε* is low and *R*_0_(*v*) is greater than unity, the disease may not be eradicated even if the vaccine coverage *v* is high. The epidemiological implication is that high vaccine efficacy and vaccination coverage will drastically reduce the number of secondary infections in the community. This result also agrees with the conclusion from Figure 2. The graphical representation (contour plots) of *R*_0_(*v*) in the parameter space (*v*, *τ*) is similar to Figure 14, and this tends to suggest that the impact of the vaccine efficacy is similar to the effect of treatment on the initial disease prevalence.

The article "A Mathematical Model of COVID-19 with Vaccination and Treatment" was published in 2021. Journal: Comput Math Methods Med.

Partial rank correlation describes the relationship between two variables while at the same time removing the effects of several other variables from the relationship [65, 66]. We perform sensitivity analysis by employing the partial rank correlation coefficients (PRCCs) and the Latin hypercube scheme to identify the impact of each model parameters on the initial disease transmission *R*_0_(*v*). PRCCs showing the effect of varying the input parameters on the effective reproduction number *R*_0_(*v*) are shown in Figure 15. All parameters with positive PRCCs will result in an increase on the number of initial disease transmission, while an increase in parameters with negative PRCCs will result in a reduction of *R*_0_(*v*). By exploring Figure 15, the most influential parameters can be identified. Model parameters that should be targeted to reduce the spread of the disease are the effective contact rate *b*, the infection reduction (vaccine efficacy) of vaccinated individuals *ε*, the fraction of exposed individuals who develop symptoms, and, respectively, the exit rates from the exposed and the asymptomatic classes *σ* and *ϕ*.

Figures 16 depicts the impact of the effective contact rate *b* and the vaccine efficacy on the effective reproduction number *R*_0_(*v*). As expected, to reduce the value of *R*_0_(*v*) below unity, the effective contact rate must be very low, almost irrespective of the vaccine efficacy. That is, despite the availability of vaccines, care-free mixing should continue to be monitored to avoid excessive number of contacts. Similarly, Figure 17 indicates that irrespective of the treatment rate, effective contact rate should be minimized to mitigate the spread of COVID-19 in the population.

## 6. Conclusion

We formulated a deterministic model of the transmission dynamics of COVID-19 with an imperfect vaccine. The model is theoretically analyzed; its effective and basic reproduction numbers are derived. The disease-free equilibrium is globally asymptotically stable, and the disease could be eradicated when the reproduction number is below unity. The critical vaccination threshold is derived, and it is noted that if the vaccine efficacy is low and the disease reproduction number is high, the disease may not be eradicated even if a large proportion of the population is vaccinated. That is, additional efforts will be needed to reduce *R*_0_(*v*) below unity even if vaccine coverage is high.

We then introduce into model system 1 time-dependent control variables *u*_1_(*t*) representing vaccination and *u*_2_(*t*) representing treatment of hospitalized individuals and applied the Pontryagin maximum principle to determine the optimal control strategy for mitigating the spread of the disease. We analytically derived the optimality conditions for disease eradication. The model fits quite well the observed daily data from Senegal early COVID-19 epidemic. Numerical simulations of the optimal control of the full model are carried out using a set of model parameter values. Numerical simulations indicate that COVID-19 can be controlled in the community with the implementation of vaccination and treatment. While our results suggest that vaccination and treatment are very effective in mitigating the spread of COVID-19, more efforts are needed to eradicate the disease. Thus, a combination of or concurrently applying personal protection/preventive measures (nonpharmaceutical public health interventions) such as face masks, hand washing, and social distancing should continue to be encouraged.

The article "A Mathematical Model of COVID-19 with Vaccination and Treatment" was published in 2021. Journal: Comput Math Methods Med.

Finally, we performed a sensitivity analysis using the partial rank correlation coefficient in conjunction with the Latin hypercube sampling technique, to identify the model parameters that significantly influence the initial disease transmission *R*_0_(*v*). Early identification of model parameters with greater influence on disease transmission is important to inform policy decision on which parameters to focus either for data collection or to mitigate the spread of the disease.

This study is not exhaustive, and future studies could investigate the impact of both therapeutic and (adherence to) nontherapeutic measures on the dynamics of COVID-19.

## Figures and Tables

**Figure 1:** Compartment diagram of the human component of the model.

**Figure 2:** Graphical representation of *ε*^∗^(*ℛ*_0_).

**Figure 3:** Graphical representation of *v*^∗^(*ℛ*_0_).

**Figure 4:** Endemic equilibrium regions when *R*_0_(*v*) > 1 in the (*ω*_*I*_, *ω*_*A*_) space.

**Figure 5:** Model fit with cumulative daily COVID-19 cases in Senegal, 29 March–29 April 2021.

**Figure 6:** Profile of *S*, *V*, *E*, and *I* without saturation.

**Figure 7:** Profile of *S*, *V*, *E*, and *I* with saturation.

**Figure 8:** Dynamics of the vaccinated class *V*.

**Figure 9:** Dynamics of the exposed class *E*.

**Figure 10:** Dynamics of the asymptomatic class *A*.

**Figure 11:** Dynamics of the infected class *I*.

**Figure 12:** Dynamics of the hospitalized class *H*.

**Figure 13:** Controls *u*_1_(*t*) and *u*_2_(*t*).

**Figure 14:** Contour plot of *R*_0_(*v*) with respect to vaccine coverage *v* and efficacy *ε*.

**Figure 15:** PRCCs showing the effect of varying the input parameters on *R*_0_(*v*).

**Figure 16:** Contour plot of *R*_0_(*v*) with respect to effective contact rate *b* and vaccine efficacy *ε*.

The article "A Mathematical Model of COVID-19 with Vaccination and Treatment" was published in 2021. Journal: Comput Math Methods Med.

**Figure 17:** Contour plot of *R*_0_(*v*) with respect to effective contact rate *b* and treatment rate *τ*.

**Table 1:** Model parameter values and source.

Parameter	Description	Value	Reference
*Π*	Recruitment rate of individuals into the population	$\frac{10000}{59\times 365}$	[26, 38]
*p*	Proportion of recruited individuals who are vaccinated	0.0001	Assumed
*v*	Vaccination rate	0.4	Assumed
*ω*_*A*_	Reduction in the transmission from asymptomatic	0.3	[39]
*ω*_*I*_	Increase in the transmission from symptomatic	1.8	Assumed
*ω*_*H*_	Reduction in the transmission from hospitalized	0.3	Assumed
*μ*	Natural death rate	$\frac{1}{59\times 365}$	[26, 38]
*δ*	Disease-induced death rate	0.018	[40, 41]
*ε*	Infection reduction of vaccinated individuals	0.8	Assumed
*σ*	Exit rate from the exposed class	0.13	[9]
*γ*	Exit rate from the infectious class	0.0833	[41]
*κ*	Proportion of infectious who recover naturally	0.05	[42]
*ψ*	Fraction of exposed who become infected	0.7	[39]
*b*	Effective contact rate	1.12	[41]
*τ*	Recovery rate of hospitalized individuals	0.0701	[40]
*ϕ*	Proportion of asymptomatic who recover naturally	0.14	[9]
*λ*	Exit rate from the asymptomatic class	0.13978	[39, 41]
*η*	Rate at which individuals lose immunity	0.011	[19]

## Data Availability

There are no underlying data.

## Appendix

### A. Expressions *P*_1_ and *P*_2_

Expressions of the coefficients *P*_1_ and *P*_2_ of quadratic equation (24), with *ε*_1_ = 1 − *ε* and *p*_1_ = 1 − *p*.

(A.1) $$\begin{array}{c} P_{1}=b\varepsilon_{1}g_{7}\gamma \kappa_{1}l\mu \omega_{H}p\phi_{1}\psi_{1}\sigma +b\varepsilon_{1}g_{7}\gamma \kappa_{1}l\mu \omega_{H}p_{1}\phi_{1}\psi_{1}\sigma +b\varepsilon_{1}g_{5}g_{7}\gamma \kappa_{1}\mu \omega_{H}p\psi \sigma +b\varepsilon_{1}g_{5}g_{7}\gamma \kappa_{1}\mu \omega_{H}p_{1}\psi \sigma +\delta \varepsilon_{1}g_{1}g_{7}\gamma \kappa_{1}lp\phi_{1}\psi_{1}\sigma +b\varepsilon_{1}g_{6}g_{7}l\mu \omega_{I}p\phi_{1}\psi_{1}\sigma +b\varepsilon_{1}g_{6}g_{7}l\mu \omega_{I}p_{1}\phi_{1}\psi_{1}\sigma +\delta \varepsilon_{1}g_{7}\gamma \kappa_{1}lp_{1}\phi_{1}\psi_{1}\sigma v+\delta \varepsilon_{1}g_{1}g_{5}g_{7}\gamma \kappa_{1}p\psi \sigma +b\varepsilon_{1}g_{5}g_{6}g_{7}\mu \omega_{I}p\psi \sigma +b\varepsilon_{1}g_{5}g_{6}g_{7}\mu \omega_{I}p_{1}\psi \sigma +b\varepsilon_{1}g_{4}g_{6}g_{7}\mu \omega_{A}p\psi_{1}\sigma +b\varepsilon_{1}g_{4}g_{6}g_{7}\mu \omega_{A}p_{1}\psi_{1}\sigma +\delta \varepsilon_{1}g_{1}g_{6}g_{7}lp\phi_{1}\psi_{1}\sigma +\delta g_{2}g_{7}\gamma \kappa_{1}lp_{1}\phi_{1}\psi_{1}\sigma +\delta \varepsilon_{1}g_{5}g_{7}\gamma \kappa_{1}p_{1}\psi \sigma v+\varepsilon_{1}\eta g_{6}\gamma \kappa l\phi_{1}\psi_{1}\sigma v+\delta \varepsilon_{1}g_{6}g_{7}lp_{1}\phi_{1}\psi_{1}\sigma v+\varepsilon_{1}\eta \gamma \kappa_{1}l\phi_{1}\psi_{1}\sigma \tau v+\delta \varepsilon_{1}g_{1}g_{5}g_{6}g_{7}p\psi \sigma +\delta g_{2}g_{5}g_{7}\gamma \kappa_{1}p_{1}\psi \sigma +\eta g_{2}g_{6}\gamma \kappa l\phi_{1}\psi_{1}\sigma +\delta g_{2}g_{6}g_{7}lp_{1}\phi_{1}\psi_{1}\sigma +\eta g_{2}\gamma \kappa_{1}l\phi_{1}\psi_{1}\sigma \tau +\varepsilon_{1}\eta g_{5}g_{6}\gamma \kappa \psi \sigma v+\delta \varepsilon_{1}g_{5}g_{6}g_{7}p_{1}\psi \sigma v+\varepsilon_{1}\eta g_{4}g_{6}l\phi \psi_{1}\sigma v+\varepsilon_{1}\eta g_{5}\gamma \kappa_{1}\psi \sigma \tau v+\eta g_{2}g_{5}g_{6}\gamma \kappa \psi \sigma +\delta g_{2}g_{5}g_{6}g_{7}p_{1}\psi \sigma +\eta g_{2}g_{4}g_{6}l\phi \psi_{1}\sigma +\eta g_{2}g_{5}\gamma \kappa_{1}\psi \sigma \tau -\varepsilon_{1}g_{1}g_{3}g_{4}g_{5}g_{6}g_{7}-g_{2}g_{3}g_{4}g_{5}g_{6}g_{7},\\ P_{2}=\delta \varepsilon_{1}g_{7}\gamma \kappa_{1}lp\phi_{1}\psi_{1}\sigma +\delta \varepsilon_{1}g_{7}\gamma \kappa_{1}lp_{1}\phi_{1}\psi_{1}\sigma +\delta \varepsilon_{1}g_{5}g_{7}\gamma \kappa_{1}p\psi \sigma +\delta \varepsilon_{1}g_{5}g_{7}\gamma \kappa_{1}p_{1}\psi \sigma +\varepsilon_{1}\eta g_{6}\gamma \kappa l\phi_{1}\psi_{1}\sigma +\delta \varepsilon_{1}g_{6}g_{7}lp\phi_{1}\psi_{1}\sigma +\delta \varepsilon_{1}g_{6}g_{7}lp_{1}\phi_{1}\psi_{1}\sigma +\varepsilon_{1}\eta \gamma \kappa_{1}l\phi_{1}\psi_{1}\sigma \tau +\varepsilon_{1}\eta g_{5}g_{6}\gamma \kappa \psi \sigma +\delta \varepsilon_{1}g_{5}g_{6}g_{7}p\psi \sigma +\delta \varepsilon_{1}g_{5}g_{6}g_{7}p_{1}\psi \sigma +\varepsilon_{1}\eta g_{4}g_{6}l\phi \psi_{1}\sigma +\varepsilon_{1}\eta g_{5}\gamma \kappa_{1}\psi \sigma \tau -\varepsilon_{1}g_{3}g_{4}g_{5}g_{6}g_{7}. \end{array}$$
